This article has been retracted.

# MicroRNA-330-3p promotes cell invasion and metastasis in non-small cell lung cancer through GRIA3 by activating MAPK/ERK signaling pathway

**DOI:** 10.1186/s13045-017-0493-0

**Published:** 2017-06-19

**Authors:** Chun-Hua Wei, Gang Wu, Qian Cai, Xi-Can Gao, Fan Tong, Rui Zhou, Rui-Guang Zhang, Ji-Hua Dong, Yu Hu, Xiao-Rong Dong

**Affiliations:** 1 Cancer Center, Union Hospital, Tongji Medical College, Huazhong University of Science and Technology, 1277 JieFang Avenue, Wuhan, 430022 People’s Republic of China; 2 Experimental Center, Union Hospital, Tongji Medical College, Huazhong University of Science and Technology, 1277, JieFang Avenue, Wuhan, 430022 People’s Republic of China; 3 Institute of Hematology, Union Hospital, Tongji Medical College, Huazhong University of Science and Technology, 1277 JieFang Avenue, Wuhan, 430022 People’s Republic of China

**Keywords:** miR-330-3p, NSCLC, Invasion and metastasis, GRIA3, DNA methyltransferase, MAPK/ERK signaling

## Abstract

**Background:**

Brain metastasis (BM) is associated with poor prognosis in patients with non-small cell lung cancer (NSCLC). Recent studies demonstrated that microRNA-330-3p (miR-330-3p) was involved in NSCLC brain metastasis (BM). However, the exact parts played by miR-330-3p in BM of NSCLC remain unknown. Discovery and development of biomarkers and elucidation of the mechanism underlying BM in NSCLC is critical for effective prophylactic interventions. Here, we evaluated the expression and biological effects of miR-330-3p in NSCLC cells and explored the underlying mechanism of miR-330-3p in promoting cell migration and invasion in NSCLC.

**Methods:**

Stable over-expression and knockdown of miR-330-3p in NSCLC cells was constructed with lentivirus. Expression levels of miR-330-3p in NSCLC cells were quantified by quantitive real-time PCR (qRT-PCR). The effects of miR-330-3p on NSCLC cells were investigated using assays of cell viability, migration, invasion, cell cycle, apoptosis, western blotting, immunohistochemical, and immunofluorescence staining. A xenograft nude mouse model and in situ brain metastasis model were used to observe tumor growth and brain metastasis. The potential target of miR-330-3p in NSCLC cells was explored using the luciferase reporter assay, qRT-PCR, and western blotting. The miR-330-3p targets were identified using bioinformatics analysis and verified by luciferase reporter assay. The correlation between GRIA3 and DNA methyltransferase (DNMT) 1 and DNMT3A was tested by RT-PCR, western blotting, and co-immunoprecipitation (IP).

**Results:**

miR-330-3p was significantly up-regulated in NSCLC cell lines. MTT assay, transwell migration, and invasion assays showed that miR-330-3p promoted the growth, migration, and invasion of NSCLC cells in vitro and induced tumor growth and metastasis in vivo. Luciferase reporter assays showed that GRIA3 was a target of miR-330-3p. qRT-PCR and western blotting exhibited that miR-330-3p promoted the growth, invasion, and migration of NSCLC cells by activating mitogen-activated protein kinase (MAPK)/extracellular-regulated protein kinases (ERK) signaling pathway. Furthermore, miR-330-3p up-regulated the total DNA methylation in NSCLC cells, and co-IP-demonstrated GRIA3 was directly related with DNMT1 and DNMT3A.

**Conclusions:**

miR-330-3p promoted the progression of NSCLC and might be a potential target for the further research of NSCLC brain metastasis.

**Electronic supplementary material:**

The online version of this article (doi:10.1186/s13045-017-0493-0) contains supplementary material, which is available to authorized users.

## Background

Lung cancer is the first leading cause of cancer-related deaths [1, 2], and non-small cell lung cancer (NSCLC) accounted for about 88% of primary lung malignancies [3–5]. Brain metastasis (BM) developed in approximately 25% of these patients [6]. BM causes significant neurologic, cognitive, and emotional consequences [7], and negatively impacts survival [8]. Previous categorizations of NSCLC in terms of BM are not satisfactory. Moreover, to date, no effective measures have been available to reduce the risk of BM in NSCLC patients.

Therefore, a good classification of NSCLC in terms of BM is needed for patient stratification. Molecular biomarkers may help, but their use is limited since they entail adequate quality tumor tissues collected in a standardized fashion for genomic profiling. Recently, microRNAs (miRNAs) have been utilized for the characterization of tumors [9, 10]. miRNAs are small non-coding RNAs of 18–25 nucleotides that might impact various stages of development and progression of cancer [11, 12]. By complementary base-pairing, miRNAs bind to sequences in the 3′-untranslated region (3′-UTR) of target mRNAs, resulting in translation inhibition or degradation of the target mRNAs [13, 14]. It has been reported that miRNAs can function as oncogenes or tumor suppressors [15–17].

Hypermethylation is responsible for the silencing of tumor suppressor genes (TSGs) involved in lung carcinogenesis, such as CDKN2A [18], CDH13 [18], FHIT [19], WWOX [19, 20], CDH1 [21], and RASSF1A [21]. Specific alterations in DNA methylation patterns are hallmarks of human diseases and therefore could serve as specific targets for cancer treatment [22, 23]. Aberrant promoter hypermethylation of CpG islands associated with tumor suppressor genes can lead to transcriptional silencing and result in tumor development [24, 25]. Methylation is controlled by DNA methyltransferases (DNMTs). Three catalytically active DNMTs have been identified in mammals, DNMT1, DNMT3A, and DNMT3B [26]. The levels of DNMT1, DNMT3A, and DNMT3B mRNA were reportedly elevated in various malignancies, including hepatic, prostate, colorectal, and breast tumors [27–30]. In lung squamous cell carcinomas, elevated DNMT1 expression has been shown to be indicative of a poorer prognosis, and elevated expression of both DNMT1 and DNMT3B have been demonstrated to be associated with hypermethylation of TSG promoters [31].

Previous studies exhibited that miR-330-3p was up-regulated in patients with prostate cancer and primary plasma cell leukemia [32, 33]. Recent studies demonstrated that miR-330-3p expression was increased in NSCLC patient tissues, and miR-330-3p was also involved in NSCLC brain metastasis (BM) [34]. These studies indicated that dysregulated miR-330-3p expression might also play an important role in the development and metastasis of NSCLC. However, the exact parts played by miR-330-3p in BM of NSCLC remained unknown.

In this study, we examined the oncogenic role of miR-330-3p and epigenetic regulation in NSCLC. We further investigated if miR-330-3p directly targeted GRIA3 by activating MAPK/ERK pathway and its correlation with both DNMT1 and DNMT3A.

## Methods

### Patient samples

Study subjects were 122 patients with histologically confirmed NSCLC (using AJCC criteria) receiving treatment during a period from January 2012 to December 2013. This study was approved by the Institutional Review Board of Huazhong University of Science and Technology (no. IORG0003571). Written informed consent was obtained from each patient. BM was established by certified oncologists based on whole brain magnetic resonance imaging (MRI). Fresh lung tumor tissues were obtained with biopsy and frozen in liquid nitrogen, then stored at −80 °C before RNA extraction. A 5-ml peripheral blood sample from each patient was drawn into a purple-top tube, processed for serum extraction centrifuged 3000rpm for 15 min within 2 h, and then experienced DNA extraction for measurement of global DNA methylation levels. Blood and tissue samples were collected prior to systemic chemotherapy or surgery for patients. Tumor EGFR mutation status in exons 18–21 was determined by examining DNA extracted from formalin-fixed, paraffin-embedded archival tumor tissues on an amplification refractory mutation system (ARMS). General data, including demographic information and smoking status, are summarized in Additional file 1: Table S1.

### Cell lines and culture conditions

Non-small cell lung cancer cells A549, HCC827, H460, PC-9, and H1975 were obtained from the American Type Culture Collection (ATCC, Manassas, VA, USA). The normal human bronchial epithelial cell line BEAS-2B was obtained from Shanghai Cancer Institute. Cells were propagated in RPMI 1640 medium (Gibco, Grand Island, NY, USA) supplemented with 10% fetal bovine serum (Gibco), and antibiotics (100 units/ml penicillin and 100 μg/ml streptomycin). Human umbilical vein endothelial cells (HUVECs) were established as previously described [35].

### Antibodies

Human anti-p-ERK, anti-ERK, anti-AKT, anti-p-AKT, and anti-caspase3 were purchased from Cell Signaling Technology (Danvers, MA, USA). Human anti-Bcl-2, anti-cyclin D1, anti-GRIA3, anti-PCNA, anti-Bax, anti-CD34, anti-DNMT1, anti-DNMT3A, and anti-DNMT3B were from Abcam (Cambridge, MA, UK). Human anti-VEGFA was procured from Santa Cruz Biotechnology (Santa Cruz, CA, USA). Bound primary antibodies were detected with goat anti-mouse antibody or goat anti-rabbit antibody (Sigma, St. Louis, MO, USA). Alexa Fluort 488-conjugated goat anti-mouse secondary antibodies were used for immunofluorescence staining.

### RNA extraction and quantitative reverse transcription-polymerase chain reaction (qRT-PCR)

The total RNA from cells was extracted with the mirVana miRNA isolation kit (Ambion, USA) according to the manufacturer’s protocol. The cDNA was synthesized from total RNA using PrimeScript™ RT Reagent Kit with miRNAs specific RT primers (Applied Biosystems, Waltham, MA) (Takara, Dalian, China) in a total reaction volume of 10 μl in TPersonal Thermocycler (Biometra, Göttingen, Germany) by following the manufacturer’s instructions. Then, miRNA cDNA was quantified using SYBR Premix Ex Taq kit (Takara, Dalian, China) in a 20-μl reaction system (Applied Biosystems, Foster city, CA). Expression data were uniformly normalized to U6, serving as the internal control. For mRNA dosage studies, complementary DNA was obtained with PrimeScript RT reagent Kit (Takara, Dalian, China) and then used as template to quantify DNMT1, DNMT3A, DNMT3B, and GRIA3 levels by SYBR Green RT-PCR Kit (Takara, Dalian, China). The relative expression levels were evaluated by using the 2^−∆∆Ct^ method.

### Construction of stable lentiviral clones

Lentiviral constructs expressing GFP (Green Fluorescent protein)-empty vector (NC-LV), GFP vector over-expressing miR-330-3p (OE-miR-330-3p-LV), or GFP vector knocking down miR-330-3p (anti-miR-330-3p-LV) were obtained from Systems Biosciences Inc., (Mountain View, CA). Virus production and cell transduction in H460 and H1975 cells were performed as reported [36] and selected with puromycin (1 μg/ml), and for in vitro experiments, cells were flow-cytometrically sorted to maintain a GFP positivity rate >95%.

### Western blotting and immunoprecipitation

Western blotting and immunoprecipitation were performed as previously reported [37]. Briefly, cells were lysed in MCLB, and clarified lysates were resolved by SDS-PAGE gel and transferred to poly-vinylidene difluoride membranes (Millipore, Billerica, MA, USA), then the membranes were blocked with 5% skimmed-milk powder in Tris-buffered saline with Tween-20 (TBS-T), incubated with the primary antibodies at 4 °C overnight, and then incubated with the secondary antibodies. The bands were detected by ECL detection reagents (Beyotime Biotechnology, Shanghai, China), and GAPDH was used as a loading control.

For immunoprecipitation, to investigate the interaction between DNMT1, DNMT3A, DNMT3B, and GRIA3 at the endogenous level, H460 and H1975 cells at 80–90% confluence were washed with ice-cold PBS three times before being lysed in IP lysis buffer. Then, the lysates were incubated with anti-DNMT1, anti-DNMT3A, or anti-DNMT3B antibodies separately overnight at 4 °C. Protein A/G-agarose beads were added for 2 h or overnight. The beads were collected and washed with lysis buffer for three times. The precipitated proteins were eluted and denatured in 2 × SDS loading buffer and analyzed by western blotting.

### Proliferation, apoptosis, and cell cycle assays

Cell proliferation was determined using MTT assay according to the manufacturer’s instructions. The absorbance was read at 450 nm on a multimode plate-reader (PerkinElmer, USA).

Cells in early and late apoptotic stages were quantified using an Annexin V-APC/PE double staining assay. Cells were collected and resuspended in 500 μL binding buffer at 1 × 10^6^ cells/ml, followed by staining with 5 μL Annexin V and 5 μL PE in the dark at room temperature for 15 min. Stained cells were immediately examined using a FACS flow cytometry analyzer (Beckman Coulter) with wavelength emission filters of 488–530 nm for the green fluorescence of Annexin V (FL1) and of 488–630 nm for the red fluorescence of PI (FL2).

For cell cycle assay, 3 × 10^5^ cells/well was seeded into a 6-well plate. After 24 h incubation, the cells were collected and fixed with 75% cold ethanol (1 mL PBS and 3 mL absolute ethanol) at −20 °C overnight. After that, the cells was incubated with 200 μL RNase A (1 mg/mL) and 500 μL propidium iodide (PI, 100 μg/mL) for 30 min at room temperature in the dark and analyzed using the FACScan flow cytometer (Becton Dickinson, Franklin Lakes, NJ, USA). The data were analyzed with ModFitLT V2.0 software (Becton Dickinson).

All experiments were performed for three independent times.

### DNA extraction and measurement of global DNA methylation levels

The genomic DNA of peripheral whole blood and transfected H460 and H1975 cells were isolated by DNeasy blood and tissue kit (Qiagen, Hilden, Germany). Global DNA methylation levels were assessed by Methylflash Methylated DNA Quantification Kit (Epigentek, Farmingdale, NY, USA) in accordance with the manufacturer’s protocol.

### Wound healing, migration, and invasion assays

For the wound healing assay, transfected H460 and H1975 cells were seeded into 6-well plates and subjected to serum starvation for 24 h in serum-free media. Afterwards, an artificial wound was created in the confluent cell monolayer of cells. Photographs were taken at 0, 24, and 48 h using an inverted microscope (Olympus, Japan). Migration and invasion assays were conducted in Transwell chambers (Costar, Corning Inc., NY, USA) coated without or with Matrigel (BD Biosciences) on the upper surface of the 8-μm (pore size) membrane. Briefly, transfected H460 and H1975 cells were harvested, suspended in serum-free medium, and plated into the upper chamber for the migration or invasion assays, respectively, and media supplemented with 10% FBS were placed into the lower chamber. After 24 h incubation, the cells that had migrated or invaded through the membrane to the lower surface were fixed, stained, and counted under an inverted microscope (Olympus, Tokyo, Japan).

### Tube formation assay

Matrigel (50 μL/well, BD) was added to 96-well plates and polymerized for 2 h at 37 °C. Cells (2–3 × 10^4^ per well) were added and cultured for 6–8 h in serum-free medium prior to image capture under a microscope at ×100 magnifications (Olympus). The tube number of branches (the branching points were parts of the skeleton where three or more tubes converged) and number of loops (a loop was an area of the background enclosed or virtually enclosed by the tubular structure) was counted.

### Collection of CM

Transfected and control H460 and H1975 cells were seeded onto 6-well plates at 2 × 10^6^/ml in RPMI-1640 supplemented with 2% fetal bovine serum. After culture for 24 h, the supernatant was collected and centrifuged at 1200 and 12000rpm respectively for 10 min to remove cell debris.

### In vitro angiogenesis assays plus co-culture with HUVECs

Cell invasion and tube formation assays were performed in the presence of conditioned medium (CM) obtained from stably transfected and control H460 and H1975 cells. 5 × 10^5^ or 2 × 10^4^ HUVEC cells were suspended in CM and plated into the upper chamber for the migration assay or into the 96-well plate for the tube formation assay as previously described [38].

### Luciferase reporter assay

3′-UTR of GRIA3 predicted to interact with miR-330-3p were amplified from human genomic DNA and cloned downstream of the firefly luciferase gene in pMIR-REPORT (Promega, Madison, WI). The construct was designated wild-type (Wt) 3′-UTR. To construct mutant vectors, putative miR-330-3p binding sites in GRIA3 3′-UTR were mutated using Quick Change Site-Direct Mutagenesis Kit (Stratagene, La Jolla, CA, USA). All inserts were sequenced to verify the mutations. Cells were harvested 48 h after co-transfection of miRNA with reporter vector and assayed with Dual Luciferase Assay (Promega) according to the manufacturer’s protocol.

### Xenograft model in nude mice and bioluminescence imaging

Female BALB/c nude mice aged 4–6 weeks were purchased from the Beijing Hua Fukang Bioscience Company (Beijing, China) and were housed and monitored in a pathogen-free environment. 4 × 10^6^ H460 and H1975 cells that stably over-expressed or knockdown miR-330-3p, negative control, and empty lentivirus were suspended in 100 μl PBS and then subcutaneously injected into the right collar of the nude mice (*n* = 5 for each group). Tumor size was measured every 3 days, and tumor volume was calculated using the formula *V* = 0.5 × a × b^2^, where *a* and *b* represented the longer and shorter tumor diameters, respectively. Four weeks later, tumor burdens were evaluated on a luminescent image analyzer (Caliper IVIS Lumina XR, LifeSciences, USA).

### Brain metastatic xenografts

Female nude mice (5–6 weeks of age) were purchased from Beijing Hua Fukang Bioscience Company (Beijing, China). For brain injection, the head of the mouse was fixed with a stereotactic apparatus and a 2- to 3-mm incision was made in the skin along the cranial midline. The injection needle was inserted 2.0 mm to the right and 0.5 mm anterior of the bregma. Roughly 10 μL of transfected H460 and H1975 cell suspensions, at a concentration of 3 × 10^7^ cells/mL in PBS, was injected into the brain parenchyma using a 2.0 mm microsyringe to a depth of 3.5 mm in the right frontal lobe of brain (*n* = 5 for each group). MRI scanner for mice was used to assess tumor burdens 25 days after injection.

### Immunohistochemical and immunofluorescence staining

Protein expression was immunohistochemically determined. Briefly, 5-μm serial sections were dewaxed in xylene and rehydrated through graded alcohols. Endogenous peroxidases were blocked (3% H_2_O_2_, 30 min), and antigens retrieved by microwaving slides. After cooling and washing, slides were blocked with goat serum (1:10; Zymed antibody diluent; 30 min). The sections were then incubated with primary antibodies at 4 °C overnight and then incubated with HRP-conjugated secondary antibodies followed by the Liquid DAB Substrate Chromogen System according to the manufacturer’s instructions. The sections were examined under a fluorescence microscope (Olympus).

### Statistical analysis

In general, unpaired two-tailed Student *t* test and one-way ANOVA were used to make inter-group comparison. The Kaplan-Meier method was used to estimate overall survival. All statistical analyses were performed with SPSS (version 16.0) and GraphPad (Version 5.0). All results were presented as mean ± SD (standard deviation) with a *P* value < 0.05 considered statistically significant.

## Results

### Up-regulation of miR-330-3p in NSCLC cell lines and BM+ patients

Our result showed that miR-330-3p was expressed in the normal human bronchial epithelial cell line BEAS-2B, and five NSCLC cell lines, including A549, H460, HCC827, H1975, and PC-9 cells. miR-330-3p expression in those NSCLC cell lines was significantly higher than in BEAS-2B (*P* < 0.001, Fig. 1a). miR-330-3p expression levels were then evaluated in a series of 122 NSCLC primary lung tissue samples, using qRT-PCR, and were found to be significantly up-regulated in subjects with BM compared to subjects without BM upon diagnosis (*P* = 0.006, Fig. 1b). In this study, H460 and H1975 cells were used for further study. For each cell line (H460 or H1975), the cells were transfected separately with empty lentivirus (NC-LV), lentivirus over-expressing miR-330-3p (OE-miR-330-3p-LV), and miR-330-3p-knockdown lentivirus (anti-miR-330-3p-LV). Cells not subjected to the lentivirus transfection were included in experiments as normal controls (NC). Transfection was verified by immunofluorescence staining (Fig. 1c) and qRT-PCR (Fig. 1d). It was found that cells were flow-cytometrically sorted to maintain a GFP positivity rate >95% by immunofluorescence staining for in vitro experiments.

**Fig. 1:** Up-regulation of miR-330-3p in NSCLC cell lines and stably transfected H460 and H975 cells. **a** miR-330-3p expression was up-regulated in NSCLC cell lines when compared with normal pneumonocytes cells (BEAS-2B). **b** After stable transfection, RNA was extracted and the miR-330-3p level was determined by qRT-PCR analysis. The amount of miR-330-3p was normalized to U6. **c** Green fluorescent protein (GFP) expression after H460 and H1975 cells transfection with lentivirus. Transfection efficiency was assessed by immunofluorescence staining (original magnification ×100). *NC* cells not subjected to viral transfection, *NC-LV* cells transfected with empty lentivirus, *OE-miR-330-3p-LV* cells transfected with lentivirus over-expressing miR-330-3p, *anti-miR-330-3p-LV* cells transfected with lentivirus knocking down miR-330-3p. Mean ± SD values of three independent experiments were shown. #*P* < 0.001 compared with Beas-2B (or NC) by one-way ANOVA

### miR-330-3p modulates proliferation, apoptosis, and cell cycle of NSCLC

The MTT assay showed that cell growth was significantly increased by over-expressed miR-330-3p 24 and 48 h after transfection (*P* < 0.05) and decreased by miR-330-3p knockdown in H460 and H1975 cells 48 h after transfection (*P* < 0.05, Fig. 2a).

**Fig. 2:** miR-330-3p regulates proliferation, cell cycle, and apoptosis of NSCLC cells. **a** The proliferative ability of H460 and H1975 cells after transfection was evaluated by MTT assay. *P < 0.05, **P < 0.01, #*P* < 0.001. **b** The cell cycle was analyzed by flow cytometry after PI staining, and the data were processed with ModFit LT program. *P < 0.05, **P < 0.01, #*P* < 0.001. **c** The apoptosis of H460 and H1975 cells was determined by Annexin V-fluorescein isothiocyanate (FITC)/7-amino-actinomycin D (7-AAD) staining. The percentages of Annexin-V-positive cells were indicated. The effect of miR-330-3p on protein expression of Bcl-2, Bax, and caspase3 was determined by western blotting. GAPDH was used as a loading control. All data were presented as mean of three independent experiments ± SD, *P* value was calculated by one-way ANOVA

PI staining revealed knocking miR-330-3p down increased the percentage of cells in the S phase and decreased the percentage of cells in the G1 phase in both H460 and H1975 cells (Fig. 2b), indicating that knocking down miR-330-3p could lead to S arrest.

Flow cytometry showed that apoptosis was inhibited in H460 cells (6.51 vs. 7.15% in cells transfected with empty vector, Fig. 2c) and H1975 cells (5.64 vs*.* 6.29%, Fig. 2c), which both over-expressed miR-330-3p. In contrast, cell apoptosis was increased by miR-330-3p knockdown in both H460 cells (46.62 vs. 7.15%, Fig. 2c) and H1975 cells (13.41 vs. 6.29%, Fig. 2c). Furthermore, detection of the expression of apoptosis-associated proteins (Bax, Bcl-2, and caspase3) exhibited that over-expressed miR-330-3p increased Bcl-2 and reduced Bax expression, and miR-330-3p knockdown increased the expression of cleaved caspase3 (Fig. 2c and Additional file 2: Figure S1).

### miR-330-3p promotes NSCLC cell migration, invasion, and angiogenesis in vitro

miR-330-3p over-expression increased the capillary-forming ability in both H460 and H1975 cells (Fig. 3a). In cells with miR-330-3p knockdown, the tubular structure was incomplete and fluffy. The wound healing assay demonstrated that the migratory ability of H460 and H1975 cells over-expressing miR-330-3p was significantly higher than that of cells transfected with empty lentivirus (Fig. 3b). Similarly, the transwell migration assay showed that miR-330-3p over-expression significantly increased the migratory ability of NSCLC cells (*P* < 0.001, Fig. 3c). Moreover, the transwell invasion assay revealed that the invasiveness of NSCLC cells over-expressing miR-330-3p was significantly higher than that of the cells transfected with the empty lentivirus (*P* < 0.05, Fig. 3d). These results indicated that miR-330-3p over-expression significantly promoted the migration, invasion, and angiogenesis of NSCLC cells in vitro.

**Fig. 3:** Over-expression of miR-330-3p induces the ability of tube formation, migration, and invasion in NSCLC cells. **a** Tube formation assay measuring proangiogenic activity in H460 and H1975 cells; tube formation was assessed using an inverted light microscope (Olympus IX71, original magnification ×100). **b** Wound-healing assays were performed to assess NSCLC cell migration. Wound closure was determined 24 h after the scratch. **c** Transwell migration assay measuring NSCLC cell migration in H460 and H1975 cells stably transfected with NC-LV, OE-miR-330-3p-LV or anti-miR-330-3p-LV, respectively. The number of migrated cells was evaluated by counting 10 random fields at ×100 magnification. **d** Transwell invasion assay was used to quantify cell invasion in a Matrigel-coated chamber. The average number of cells invading per field of view in three different experiments is plotted. *Error bars* indicate mean ± SD, a representative experiment of three was reported. *P < 0.05, **P < 0.01, #*P* < 0.001, one-way ANOVA

Culture of HUVEC cells in conditioned medium extracted from culture supernatant of H460 or H1975 cells showed that tube formation, migration, and invasion of HUVEC cells were enhanced by miR-330-3p over-expression in NSCLC cells and decreased by miR-330-3p knockdown (*P* < 0.05 for both, Fig. 4a–c). Additionally, miR-330-3p over-expression elevated the level of VEGFA expression (Fig. 4d).

**Fig. 4:** miR-330-3p promotes tube formation, migration, and invasion in HUVECs co-cultured with NSCLC cells. **a** HUVECs were seeded on top of extracellular matrix, in the presence of conditioned medium (CM). Photographs are representative of three independent experiments (original magnification ×100). **b** HUVECs were seeded in 6-well plates, in the presence of CM. Wound closure was determined 6 and 12 h after the scratch. **c** Cell invasion was evaluated using a 24-transwell chamber with 8-μm pore insert. HUVECs were seeded in the upper chamber, in the presence of CM. The migrated cells were crystal violet-stained and assessed using an inverted light microscope (original magnification ×100). CM was obtained from NC-LV, OE-miR-330-3p-LV, or anti-miR-330-3p-LV-transfected H460 and H1975 cells. **d** The expression of VEGFA in H460 and H1975 cells after different treatment by western blotting. *Error bars* indicate mean ± SD, a representative experiment of three was reported; *P < 0.05, **P < 0.01, #*P* < 0.001, *P* value was calculated by one-way ANOVA

### miR-330-3p promotes the growth of NSCLC xenograft tumors in vivo

To further explore whether ectopic expression of miR-330-3p affects tumor growth in vivo, we made a xenograft tumor model by subcutaneously injecting into the front flank of nude mice the H460 and H1975 cells stably over-expressing miR-330-3p, cells with miR-330-3p knockdown or cells transfected with empty vector. The results showed that tumors injected with miR-330-3p-knock down H460 and H1975 cells grew more slowly and were of small size as compared with the tumors injected with cells with empty vector (*P* < 0.05, Fig. 5a–c). The survival time was shorter in mice injected with H460 and H1975 cells over-expressing miR-330-3p (*P* < 0.05 vs. tumors injected with empty vector cells, Fig. 5d). Furthermore, immunohistochemical analysis revealed that miR-330-3p over-expression increased the expression of PCNA and cyclin D1 and decreased the expression of caspase3 and Bax in tumors when compared with the NC group, knocking down miR-330-3p decreased PCNA, and cyclin D1 expression and increased caspase3 and Bax expression in tumors (Fig. 6a and Additional file 3: Figure S3a–d). Immunofluorescence staining revealed that CD34 expression was down-regulated, and stained vessels were less in tumors injected with miR-330-3p-knockdown cells (Fig. 6b).

**Fig. 5:** miR-330-3p induces tumorigenesis in a xenograft mouse model. **a**, **b** H460 and H1975 cells stably transfected with NC-LV, OE-miR-330-3p-LV, or anti-miR-330-3p-LV were injected subcutaneously into nude mice. Four weeks after the injection, mice were photographed and killed. Tumor growth curves were obtained. All data were presented as mean of three independent experiments ± SD, *P < 0.05, **P < 0.01, #*P* < 0.001, one-way ANOVA test. **c** Representative bioluminescence images of tumor burden in the mice that received subcutaneous injection of indicated cells. **d** *Survival curves* represent the duration from injection until 4 weeks when mice were killed

**Fig. 6:** miR-330-3p induces tumor metastasis and angiogenesis in BM model. **a** Immunohistochemical analysis of PCNA, cylinD1, Bcl-2, Bax, caspase3, DNMT1, DNMT3A and DNMT3B expression in tissue sections of GFP-labeled tumors isolated from mice injected with H460 and H1975 cells transfected with NC-LV, OE-miR-330-3p-LV or anti-miR-330-3p-LV. A representative experiment of three was reported. *P < 0.05, **P < 0.01, #*P* < 0.001, one-way ANOVA test. **b** Representative images of CD31-positive endothelial cells in the viable tumor tissue of mice. **c** MRI analysis of metastatic tumors (*yellow arrow*) in the brain. Representative MRI of tumors is shown

### miR-330-3p promoted brain metastasis tumor growth

After cells were orthotopically implanted into the brain, general conditions (weight loss and cancerous cachexia) deteriorated much faster in mice receiving H460 or H1975 cells over-expressing miR-330-3p. MRI imaging at 25 days revealed more metastatic foci in mice receiving NSCLC cells over-expressing miR-330-3p than in those receiving cells transfected with empty vector or non-transfected cells (Fig. 6c). Most mice receiving H460 and H1975 cells with miR-330-3p knockdown did not have tumor foci (Fig. 6c). These finding suggested that miR-330-3p could promote the growth of tumors in the brain.

### GRIA3 is a direct target of miR-330-3p

Search of publicly available databases (TargetScan, miRanda, and HOCTar) revealed that GRIA3 was a potential target of miR-330-3p (Additional file 1: Table S2). GRIA3 was found to play an important role in the growth and metastasis of malignant cells [39]. Then, we constructed luciferase reporter vectors containing the wild-type or mutant miR-330-3p sequences of the GRIA3 3′-UTR, and conducted luciferase reporter assays to see whether GRIA3 is a direct target of miR-330-3p. After co-transfection with the miR-330-3p mimics, the luciferase activity of the wild-type 3′ UTR reporter gene was significantly inhibited, whereas the activity of the mutant reporter gene was not affected by the miR-330-3p mimics (*P* < 0.05, Fig. 7a), indicating that miR-330-3p could bind to the GRIA3 3′-UTR. Subsequent experiments demonstrated that over-expression of miR-330-3p significantly down-regulated the mRNA and protein expression of GRIA3 (*P* < 0.01, Fig. 7b, c). These results demonstrated that miR-330-3p could directly suppress the expression of GRIA3 in NSCLC cells by directly targeting the GRIA3 3′-UTR.

**Fig. 7:** GRIA3 is a direct target of miR-330-3p. **a** Relative luciferase activity of 293 T cells after co-transfection with wild-type (Wt) or mutant (Mt) GRIA3 3′ UTR reporter genes and miR-330-3p mimics or control. The expression of GRIA3 in H460 and H1975-transfected cells was determined by qRT-PCR (**b**) and by western blotting (**c**). **d** Transwell invasion assays of H460 and H1975 cells transfected with lentivirus either empty (NC-LV) or miR-330-3p (330-3p) followed by GRIA3 or pcDNA control (Vec) vectors. All data were presented as mean of three independent experiments ± SD. *P < 0.05, **P < 0.01, #*P* < 0.001, one-way ANOVA test

To determine the importance of the target gene in miR-330-3p-mediated functions such as invasion, we performed rescue assay where GRIA3 was over-expressed in H460 and H1975 cells with elevated miR-330-3p level. We observed that GRIA3 over-expression was able to prevent or reverse the increased invasiveness in H460 and H1975 cells caused by miR-330-3p (*P* < 0.05, Fig. 7d). These data indicated that GRIA3 was an important and direct target of miR-330-3p in regulating NSCLC cell metastasis.

### miR-330-3p promotes global DNA methylation and suppresses the expression of hypermethylated p16^INK4A^ in NSCLC cells

Emerging evidences have suggested that hypermethylation are well-established molecular alterations involved in cancer progression leading to metastasis [40, 41], it is reasonable to envision that DNA methylation can orchestrate the highly dynamic brain metastasis process. Analysis of epigenetic modifications in NSCLC showed that global DNA methylation was significantly increased in H460 and H1975 cells over-expressing miR-330-3p as compared with cells with empty vector (*P <* 0.05, Fig. 8a). Furthermore, we examined the global DNA methylation level of peripheral whole blood samples in newly diagnosed NSCLC patients with or without brain metastasis (BM+ or BM−). The global DNA methylation level was higher in BM+ than in BM− patients (*P <* 0.05, Fig. 8b, *n* = 10).

**Fig. 8:** miR-330-3p regulates DNA methylation, and GRIA3 interacts with DNMT1 and DNMT3A. Global DNA methylation changes are measured in H460 and H1975 cells transfected with NC-LV, OE-miR-330-3p-LV, or anti-miR-330-3p-LV (**a**) and tumor tissue of NSCLC patients with or without BM (*n* = 5) (**b**). **c** DNMT1, DNMT3A, and DNMT3B mRNA expression levels in H460 and H1975 cells transfected with NC-LV, OE-miR-330-3p-LV, or anti-miR-330-3p-LV were assessed by qRT-PCR. **d** DNMT1, DNMT3A, DNMT3B, and p16^INK4A^ protein expression levels are assessed by western blotting; GAPDH is used as an internal control. **e** H1975 cells were lysed with MCLB, and lysates were subjected to immunoprecipitation using anti-IgG, anti-DNMT1, DNMT3A, or anti-DNMT3B as indicated and were analyzed by western blotting. Each *bar* represents mean ± SD of triplicate samples from a representative experiment. *P < 0.05, **P < 0.01, *P* value was calculated by one-way ANOVA

Then, we analyzed the expression of p16^INK4A^ in H460 and H1975 cells to further examine the effect of DNA methylation-regulated miR-330-3p on TSGs. Re-expression of p16^INK4A^ protein was found in H460 and H1975 cells with miR-330-3p knockdown (Fig. 8d and Additional file 4: Figure S4d).

Collectively, these findings suggested that miR-330-3p could inactivate TSGs in tumorigenesis by DNA hypermethylation, whereas miR-330-3p inhibition could partially reverted aberrant methylation in cancer cells.

### miR-330-3p is directly relevant to DNMT1 and DNMT3A in NSCLC cells

qRT-PCR and western blotting revealed that miR-330-3p over-expression was found to markedly increase the expression of DNMT1 and DNMT3A (*P <* 0.05, Fig. 8c, d and Additional file 4: Figure S4a, b). Nonetheless, neither miR-330-3p over-expression nor its knockdown significantly changed DNMT3B expression at both mRNA and protein levels in H460 and H1975 cells (Fig. 8c, d and Additional file 4: Figure S4c). Moreover, immunohistochemical analysis revealed that miR-330-3p over-expression increased the expression of DNMT1 and DNMT3A in tumors when compared with the NC group, knocking down miR-330-3p decreased DNMT1 and DNMT3A expression in tumors (Fig. 6a and Additional file 3: Figure S3e–g). Further endogenous co-IP found that GRIA3 was directly associated with DNMT1 and DNMT3A (Fig. 8e). Taken together, these findings suggested that miR-330-3p could directly regulate DNMTs expression in NSCLC cells.

### MAPK/MEK/ERK signaling

Western blotting showed that miR-330-3p over-expression increased p-AKT and p-ERK in H460 and H1975 cells (Fig. 9a, b). Treatment with U0126, a MEK1/2 inhibitor, increased GRIA3 level in H460 and H1975 cells over-expressing miR-330-3p and in cells with miR-330-3p knocked down (Fig. 9a). Treatment with PI3K/AKT inhibitor LY294002 did not change GRIA3 expression (Fig. 9b). The migration and invasion of H460 and H1975 cells over-expressing miR-330-3p was inhibited by U0126 but not by LY294002 (Fig. 9c, d). These results suggested that malignant behaviors might be induced by miR-330-3p in NSCLC cells by activating MAPK/ERK pathway and down-regulating GRIA3.

**Fig. 9:** miR-330-3p played its roles in promoting invasion and metastasis of NSCLC cells through modulating the expression of GRIA3 via MAPK/ERK pathway. The expression of GRIA3 was determined by western blotting when cells were treated with MEK inhibitor (U0126) (**a**) and PI3K inhibitor (LY294002) (**b**). Representative images (*upper*) and quantification (*lower*) of the transwell migration assay (**c**) and transwell invasion assay (**d**) of H460 and H1975 cells treated with MEK inhibitor (U0126). Values are mean ± SD; a representative experiment of three was reported *P < 0.05, **P < 0.01, one-way ANOVA test

## Discussion

In NSCLC patients, brain metastasis (BM) can cause neurologic, cognitive, and emotional disorders [7]. Identifying patients at risk for BM may help to prevent the condition from further deterioration. However, previous efforts to stratify NSCLC patients in terms of risk for BM have been unsatisfactory. So far, no effective measures have been available to reduce the risk of BM in NSCLC patients. Thus, looking for the biomarkers that are accurately indicative of BM may help address the development of BM in NSCLC.

In recent years, research efforts have been directed at using microRNAs (miRNAs) to characterize tumors. In general, one miRNA appears to be able to regulate several hundreds of genes, and as a result, miRNA profiling could serve as a better classifier than gene expression profiling [42]. Previous studies have shown that miR-330-3p was up-regulated in the blood of patients with prostate cancer and primary plasma cell leukemia [32, 33]. Moreover, miR-330-3p expression was found to be increased in the tissues of NSCLC patients, and miR-330-3p was also involved in BM in NSCLC patients with its expression being 53-fold higher as compared with non-metastatic NSCLC [34, 43, 44] A recent study showed that miR-330-3p could successfully distinguish BM+ vs. BM- cases in a validation cohort of NSCLC patients [34]. The aforementioned studies indicated that dysregulated miR-330-3p expression might also play an important role in the tumorigenesis of NSCLC. However, the exact parts played by miR-330-3p in NSCLC are still poorly understood.

In this study, we found that miR-330-3p was over-expressed in NSCLC cells as compared with the normal human bronchial epithelial cells (BEAS-2B). Since migration and invasion are the key steps of tumor metastasis, we performed a migration and an invasion assay to determine the role of miR-330-3p in the metastasis of NSCLC cells (H460 and H1975 cells). Our study showed that miR-330-3p over-expression led to increased migration and invasion of H460 and H1975 cells, suggesting that miR-330-3p over-expression imparted a migratory and invasive advantage to NSCLC cells. Next, we observed that miR-330-3p over-expression could inhibit cell apoptosis and promote cell proliferation, knocking down miR-330-3p resulted in S/G_2_ arrest.

It has been reported that the level of microvessels per microscopic field has metastatic and prognostic significance in some cancers [45, 46]. In this study, we examined the role of miR-330-3p in angiogenesis both in vitro and in vivo and found that miR-330-3p substantially promoted the vascularization. Specifically, our results showed that the average microvascular density (MVD) was much higher in H460 and H1975 cells tumors over-expressing miR-330-3p than in cells with miR-330-3p knockdown. It has been well accepted that higher MVD might be a key factor for the development of brain metastasis in NSCLC patients. What is more, previous studies showed that VEGF promoted tumorigenesis via angiogenesis [47, 48]. This study confirmed that VEGF was up-regulated in the NSCLC cells over-expressing miR-330-3p. By establishing a xenograft model, we found that miR-330-3p over-expression also greatly promoted tumor formation and metastasis.

By searching three miRNA target prediction databases (TargetScan, miRanda, and HOCTar) and conducting a luciferase reporter assay, we showed that GRIA3 was a target of miR-330-3p in NSCLC cells. GRIA3 is a subunit of ionotropic glutamate receptors (AMPAR) [39] and was shown to promote tumor progression in glioma [49, 50] and pancreatic cancer [39]. In this study, western blotting and qRT-PCR demonstrated that GRIA3 level was inversely correlated with miR-330-3p expression. Since AMPAR signaling to KRAS and MAPK pathways, promoted migration and invasion of cells [51], and GRIA3 acted as an important mediator of survival, proliferation, and migration of tumor cell, which, in pancreatic cancer, are regulated by CUX1 downstream of PI3K/AKT [52], we investigated the MAPK/ERK and PI3K/AKT signaling pathways in the migration and invasion of NSCLC cells. Our results revealed that miR-330-3p over-expression increased p-ERK in both H460 and H1975 cells; however, when MEK1/2 was inhibited with U0126, a selective inhibitor, in H460 and H1975 cells, miR-330-3p over-expression decreased the expression of GRIA3. These findings suggested that miR-330-3p worked on GRIA3 via MAPK/MEK/ERK pathway to promote proliferation, invasion, and migration of NSCLC cells. Based on these findings, we were led to speculate that miR-330-3p could mediate the proliferation, migration, and invasion of tumor cells, thereby promoting BM via GRIA3.

Loss of gene transcription due to promoter hypermethylation is a crucial event in the development and progression of cancer [53]. In lung tumorigenesis, over-expression of three functional DNMTs (DNMT1, DNMT3A, and DNMT3B), which catalyze 5′ CpG methylation, might therefore be of importance for the deregulation of gene expression, especially for the deregulation of TSGs, leading to cancer formation and poor prognosis. In this study, the proteins of DNMT1 and DNMT3A were highly expressed in NSCLC cells over-expressing miR-330-3p, and the over-expression was in line with 5′ CpG hypermethylation of total DNA. Endogenous co-IP assay showed that GRIA3 bore a relation to DNMT1 and DNMT3A at endogenous levels. Taken together, miR-330-3p, acting as a promoter of NSCLC metastasis, may, by activating MAPK/ERK signaling pathway, induce 5′ CpG hypermethylation of GRIA3 and lead to the down-regulation of GRIA3 expression.

## Conclusions

In summary, this study showed that miR-330-3p promoted BM of NSCLC by enhancing cell proliferation, migration, invasion, and tumor angiogenesis. MiR-330-3p may serve as a biomarker for characterizing NSCLC patients with BM potential, and miR-330-3p might be used as a target for the treatment of NSCLC.

## Additional files

Additional file 1: Table S1. Clinical characteristics of the patients included in this study. Table S2. The sequence of predicted targetof miR-330-3p. (DOCX 17 kb)

Additional file 2: Figure S2. miR-330-3p suppresses apoptosis of NSCLC cells. a Quantitative analysis of relative protein expression for Bcl-2 detected by western blotting. b Quantitative analysis of relative protein expression for Bax detected by western blotting in each group. c Quantitative analysis of relative protein expression for cleaved caspase3 detected by western blotting in each group. All data were presented as mean of three independent experiments ± SD. *P < 0.05, **P < 0.01, #*P* < 0.001, one-way ANOVA test. (TIF 523 kb)

Additional file 3: Figure S3. Immunohistochemical analysis in tissue sections of GFP-labeled tumors isolated from mice injected with H460 and H1975 cells transfected with NC-LV, OE-miR-330-3p-LV, or anti-miR-330-3p-LV. Relative quantitative analysis of immunohistochemistry for PCNA (a), cyclinD1 (b), apoptosis-related proteins (c, d), and DNA methyltransferases (e–g). All data were presented as mean of three independent experiments ± SD. *P < 0.05, **P < 0.01, #*P* < 0.001, one-way ANOVA test. (TIF 941 kb)

Additional file 4: Figure S4. miR-330-3p is relevant to DNMT1 and DNMT3A in NSCLC cells. a DNMT1 protein expression was quantified by western blotting analysis. b Quantitative analysis of DNMT3A detected by western blotting. c DNMT3B protein expression was assessed by western blotting. d Quantitative analysis of p16^INK4A^ detected by western blotting. Error bars indicate mean ± SD for three independent experiments. *P < 0.05, **P < 0.01, #*P* < 0.001. *P* value was calculated by one-way ANOVA test. (TIF 625 kb)

## Abbreviations

3′-UTR: 3′-untranslated region
BM: Brain metastasis
CM: Conditioned medium
co-IP: Co-immunoprecipitation
DNMT: DNA methyltransferase
ERK: Extracellular regulated protein kinases
ERK1/2: Extracellular signal-regulated kinase ½
GFP: Green fluorescent protein
GRIA3: Glutamate receptor 3
HUVECs: Human umbilical vein endothelial cells
MAPK: Mitogen-activated protein kinase
miR-330-3p: MicroRNA-330-3p
miRNAs: MicroRNAs
MVD: Microvascular density
NSCLC: Non-small cell lung cancer
PCNA: Proliferating cell nuclear antigen
PI3K: Phosphoinositide 3-kinase
qRT-PCR: Quantitive real-time PCR
TSGs: Tumor suppressor genes
VEGFA: Vascular endothelial growth factor A
Wt: Wild-type
